The article "Analysis on Logistics Efficiency Measurement of New Western Land-Sea Corridor under the Background of “Double Carbon” and Ecological Environment Protection" was published in 2023. Journal: J Environ Public Health.

# Analysis on Logistics Efficiency Measurement of New Western Land-Sea Corridor under the Background of “Double Carbon” and Ecological Environment Protection

**DOI:** 10.1155/2023/8642841

**Published:** 2023-02-13

**Authors:** Tingyan Zhou, Wenxing Li

**Affiliations:** School of Economics and Management, Beijing Jiaotong University, Beijing 100044, China

## Abstract

Under the research background of ecological environment protection and “double carbon” goal, this paper applies panel data on the logistics industry from 2010 to 2019 in 12 provinces of China's new western land-sea corridor to statically measure the logistics industry's technical efficiency after taking into account the impact of different environmental elements and to analyze the dynamics trends of total factor productivity in the logistics sector. It is measured by using the three-stage SBM model and the Malmquist–Luenberger productivity index, which considers undesirable output. The findings indicate the following: (1) In the context of “double carbon,” the overall technical efficiency of the logistics sector in the new western land-sea corridor seems to be relatively low; however, the average technical efficiency of the logistics sector in the southern portion of the new western land-sea corridor does seem to be higher than that of the northern part. (2) The logistics industry's technical efficiency varies greatly by region, with locations near central China having much higher technical efficiency than remote inland areas. (3) The fundamental reason for the improvement of technical efficiency in the logistics industry is pure technical efficiency, and the driving force behind the increase in total factor productivity is technological advancement. (4) Economic development, informatization development, industrial market scale, and import and export all have a substantial influence on the logistics industry's technical efficiency. Finally, depending on the findings, policy recommendations are offered.

## 1. Introduction

With the rapid development of China's economy, the pollution and destruction of the ecological environment have been unable to make the economy sustainably developed, therefore, China has formulated the corresponding implementation of ecological protection. A major strategic objective for high-quality economic development and environmental sustainability in China is to accomplish the aim of “peak carbon dioxide emissions and carbon neutrality” [1]. During the fourteenth Five-Year Plan phase (2021–2025), the logistics industry needs to shoulder the responsibility of reducing emissions while developing at a high quality. The logistics industry's efficiency is a comprehensive indicator to measure the whole logistics operation and resource allocation in regional logistics development. In the regional coordinated development pattern based on the external environment, it is especially crucial to explore the logistics industry efficiency, enhance the allocation efficiency of input factors in the logistics industry, and enable the growth of “high quality” with “good efficiency.”

“Increase the efficiency of the logistics sector by strengthening the construction of transport infrastructure in western China, synergizing with the expansion of the Yangtze River Economic Belt,” according to the comprehensive plan for the new western land-sea corridor [2]. The new western land-sea corridor connects the Maritime Silk Road with the Overland Silk Road, offering a crucial commercial and logistical corridor for the opening up of western China's inland areas. The new western land-sea corridor's competitive development index of 113.2 in 2020 demonstrates a strong development trend as well as a considerable increase in the logistics industry's service and operational efficiency [3]. The container throughput of Beibu Gulf seaport in Guangxi has increased by 64% year-on-year, from 3.08 million TEUs in 2018 to 5.05 million TEUs in 2020. Rail-sea trains in the western area have climbed by 299 percent year-on-year, from 1,154 trains in 2018 to 4,607 trains in 2020 [4]. At the same time, with the fast expansion of the logistics sector, the energy consumption of logistics industry will increase at a high speed. Statistics on the overall energy consumption of the logistics sector in 12 provinces of the new western land-sea corridor increased from 73,272,801 tons of standard coal in 2010 to 101,375,500 tons of standard coal in 2019, with 3.67 percent average annual growth rate.

In the context of “double carbon,” can logistics sector in the new western land-sea corridor expand at an efficient and sustainable speed? Are all kinds of input resources adequately distributed and utilized? Is there a significant difference in the growth of the logistics sector among provinces in the new western land-sea corridor? This paper investigates the growth of the logistics sector along the new western land-sea corridor to show the extent to which the external environmental variables influence logistics industry's efficiency, and it serves as a reference for the improvement of logistics sector's efficiency from the perspective of rational resource allocation. Furthermore, it serves as a decision-making foundation for the construction of China's international commerce corridor with the shortest transportation time to ASEAN countries.

## 2. Literature Review

Charnes et al. [5], used data envelope analysis (DEA) to evaluate the relative efficiency of decision-making units (DMUs) with multiple inputs and multiple outputs. DEA is a nonparametric linear programming approach with a flexible calculation mechanism. It is not required to perform a certain type of production function and allows the existence of inefficiencies. Most study adopts DEA to assess the efficiency of the regional logistics sector. Tian and Li [6] utilized the DEA-Malmquist model to assess the logistics sector's total factor productivity in 30 provinces of China between 1999 and 2006 and found that there were disparities in total factor productivity and scale inefficiency among the provinces. Markovits-Somogyi and Bokor [7] employed DEA and DEA-PC to assess the logistics industry efficiency in 29 European nations, both methods are considered more appropriate after comparison. Yu and Qian [8] analyzed the logistics industry's technological efficiency in 11 provinces of the Yangtze River Economic Belt between 2006 and 2015 through the DEA-Malmquist method, concluding that it was generally not high, with the eastern area being better than the western area, and that the logistics industry's efficiency increase was primarily influenced by economic growth, informatization development, and degree of openness. Lei et al. [9] studied the technical progress index of China's 49 listed logistics businesses from 2008 to 2017 and concluded that the logistics sector's technical progress had a major beneficial influence on the skill structure of employment. Although DEA has unique advantages in measuring the input-output efficiency of DMUs, it does not account for the effect of random errors on output, which easily leads to errors in calculation results.

Stochastic frontiers analysis (SFA) is a standard representation of the parametric method with the benefit of utilizing a production function to evaluate the input-output efficiency while accounting for stochastic error. Fan and Wang [10] measured the service efficiency of 11 logistics corridors in China from 2000 to 2013 and found that the logistics corridors differed significantly in time and space, with lower service efficiency when running through western China or across eastern, central, as well as western China. Zhang et al. [11] examined the technological efficiency of low-carbon development in China's logistics sector from 2007 to 2016, and believed that the overall situation was low and the regional differences were obvious. The proportion of secondary sector in the provincial GDP and the average size of logistics enterprises have a favorable influence on the improvement of logistics industry's technical efficiency, while financial support and energy consumption have a negative influence on technical efficiency, and the impacts of environmental regulation are not obvious. Han and Liu [12] investigated the efficiency of 80 Chinese logistics listed enterprises from 2013 to 2017, concluding that total logistics company efficiency is increasing, and the average technical efficiency of enterprises in the eastern area is higher than enterprises throughout the western and central areas. Although the influence of random error is considered in the SFA model, there is no precise theoretical support when choosing the production function, and there are strict assumptions about the distribution of inefficiency terms [13].

A three-stage DEA model was proposed, which integrates the benefits of parametric and nonparametric analysis methods, excludes the effects of external environmental factors and statistical noise on efficiency evaluation, and allows measurement results to more accurately describe the internal managerial level of the decision-making unit [14]. According to Zhong [15], when the influence of external environmental factors and statistical noise are removed, the technological efficiency, pure technological efficiency, and scale efficiency of China's logistics sector change significantly. J. Zhang and J. Zhang [16] examined the logistics industry's efficiency in 31 provinces in China from 2010 to 2014 and discovered that the scale efficiency of logistics industry was increasing as a whole, but the degree of logistics operation and management restricted the logistics expansion. According to Zhang et al. [17], from 2009 to 2014, the overall logistics sector's efficiency of the New Silk Road Economic Belt at home and abroad was not high, with large differences in logistics industry's efficiency among regions being more influenced by scale efficiency. Mei et al. [18] evaluated the logistics sector efficiency in East China between 2012 and 2016 and concluded that the logistics sector was in a state of increasing scale efficiency on the whole. Increasing the retail volume of social consumer goods might enhance the logistics sector's efficiency. Yang [19] found that Jiangsu province's logistics industry performed well overall under low-carbon constraints from 2007 to 2016 and scale efficiency was the primary problem restricting the logistics industry's efficiency. Zhang et al. [20] analyzed the logistics sector's efficiency in 19 provinces of the Yangtze River Great Protection Region between 2013 and 2017 and found that the growth of the logistics sector in this area was unbalanced, with scale efficiency leading to the largest increase in technical efficiency. The three-stage DEA only evaluates the influence of desirable output on efficiency but does not consider the impact of undesirable output on efficiency. It does not objectively reflect the true level of industry management and thus measure the efficiency of the logistics industry.

Tone [21] proposed a slacks-based measure (SBM) including undesirable outputs relying on DEA improvement, thereby enhancing the scientific reliability of the efficiency measurement. Liu and Guan [22] argued that the logistics industry in China's 30 provinces was generally inefficient under low-carbon constraints from 2003 to 2014, with the inefficiencies concentrated in western China. Deng and Shen [23] evaluated the logistics industry's efficiency in 30 Chinese provinces subject to carbon emission constraints in 2016 and reported that there were significant local differences in China. The fundamental restriction to logistics development was inefficient scale, and energy structure was negatively connected to logistics sector efficiency. Zheng et al. [24] used the SBM in conjunction with hierarchical regression to measure the logistics industry's efficiency in 18 Chinese provinces bound by carbon emission constraints from 2007 to 2017, concluding that the efficiency gap across eastern and western regions had narrowed, with external variables positively influencing efficiency having shifted from the degree of openness prior to 2013 to regional economic development. Although a nonradial, nonoriented SBM with undesirable output can avoid the problems of slack and single output variable, it cannot accurately and objectively reveal the efficiency of the logistics industry without distinguishing internal managerial inefficiencies from external environmental influences and statistical noise.

In conclusion, although the three-stage DEA may remove the effects of external environment variables and statistical noise from efficiency evaluation, it cannot fully account for the slack in input-output variables and undesirable output, which leads to efficiency measurement error. The slack problem can be avoided by considering the undesirable output of the SBM model but not the interference of external environmental variables and statistical noise. Most studies have been undertaken on China as a whole, or on a specific province, or on a regional economic belt. Results vary, and systematic studies of the new western land-sea corridor are scarce. Based on this, this paper expands as follows:

1. In terms of the research methodology, the technical efficiency of the logistics industry in 7 provinces, 4 autonomous regions, and 1 municipality (henceforth referred to as 12 provinces) along the new western land-sea corridor in China from 2010 to 2019 was analyzed using a three-stage SBM model considering nonradial, nonoriented, and undesirable output. In order to complete the multidimensional extension of the study, the Malmquist–Luenberger index is used to dynamically analyze the fluctuation of total factor productivity (TFP) in the logistics sector.
2. In terms of research content, this study uses the panel data to make an empirical analysis of the logistics industry in 12 provinces of the new western land-sea corridor from 2010 to 2019, to assess the overall efficiency of the logistics sector, identify the main affecting factors, and analyze the different regional situations to expand the study of logistics industry's efficiency in less developed regions.

Figure 1 shows the research frameworks of this paper.

## 3. Methodology

### 3.1. Three-StageSlacks-Based Measure (SBM) Including Undesirable Output

#### 3.1.1. The First Stage: The Initial Slacks-Based Measure (SBM) Including Undesirable Output

Assuming the system has *n* DMUs, each of which consumes input index *x* ∈ *R*^*m*^, produce desirable output index *y*^*g*^ ∈ *R*^*s*_1_^, undesirable output index *y*^*b*^ ∈ *R*^*s*_2_^, and hypothesis matrix *X*=[*x*_1_, ⋯, *x*_*n*_] ∈ *R*^*m*×*n*^ > 0,*Y*^*g*^=[*y*_1_^*g*^, ⋯, *y*_*n*_^*g*^] ∈ *R*^*s*_1_^^×*n*^ > 0, *Y*^*b*^=[*y*_1_^*b*^, ⋯, *y*_*n*_^*b*^] ∈ *R*^*s*_2_^^×*n*^ > 0.

(1) $$\begin{array}{c} \rho =\min\frac{1-\left(1/m\right)\sum_{i=1}^{m}s_{i}^{-}/x_{i0}}{1+\left(1/s_{1}+s_{2}\right)\left(\sum_{r=1}^{s_{1}}\left(s_{r}^{g}/y_{r0}^{g}\right)+\sum_{r=1}^{s_{2}}\left(s_{r}^{b}/y_{r0}^{b}\right)\right)}\text{,}\\ subject\;to\left\{\begin{array}{l} x_{0}=X\lambda +s^{-},\\ y_{0}^{g}=Y^{g}\lambda -s^{g},\\ y_{0}^{b}=Y^{b}\lambda +s^{b},\\ s^{-}\geq 0,s^{g}\geq 0,s^{b}\geq 0,\lambda \geq 0\text{.} \end{array}\right. \end{array}$$

where *ρ* is the efficiency and 0 ≤ *ρ* ≤ 1. When *ρ*=1, *s*^−^, *s*^*g*^, *s*^*b*^ are all zero, and DMU is valid, *s*^−^ ∈ *R*^*m*^ is the input slack variables, *s*^*g*^ ∈ *R*^*s*_1_^ is the desirable output slack variable, *s*^*b*^ ∈ *R*^*s*_2_^ is the undesirable output slack variable, and *λ* ∈ *R*^*n*^ is the weight [21].

#### 3.1.2. The Second Stage: Stochastic Frontiers Analysis (SFA)

The primary purpose of the second stage is to divide the input slack variable from the first stage into three variables: internal managerial inefficiency, external environmental influences and statistical noise, and to reduce the effects of the environmental and statistical noise on efficiency evaluation.

Firstly, the dependent variables are the input slack elements obtained in the first phase, and the independent variables are the external environmental variables, which are regressed by using a Stochastic frontier analysis (SFA) to generate new input variables.

(2) $$\begin{array}{c} s_{ni}=f^{n}\left(z_{i};\beta^{n}\right)+v_{ni}+\mu_{ni},n=1,\cdots ,N,i=1,\cdots ,I, \end{array}$$

where *s*_*ni*_ is the slack variable of the ith DMU's nth input, *f*^*n*^(*z*_*i*_; *β*^*n*^) indicate the effect of external environmental variable on input slack variables, *z*_*i*_=(*z*_1*i*_, *z*_2*i*_, ⋯, *z*_*ki*_) are *k* external environmental variables, *β*^*n*^ are the parameter vectors, *v*_*ni*_ represent statistical noise, and *μ*_*ni*_ represent inefficient management.

Secondly, the SFA results are used to adjust input variables for all DMUs to a more favorable external environment and to eliminate the impact of external environmental variables and statistical noise on efficiency measurements.

(3) $$\begin{array}{c} x_{ni}^{A}=x_{ni}+\left[\max\;\left(f\left(z_{i};{\hat{\beta }}^{n}\right)\right)-f\left(z_{i};{\hat{\beta }}^{n}\right)\right]+\left[\max\left({\hat{v}}_{ni}\right)-{\hat{v}}_{ni}\right],n=1,\cdots ,N,i=1,\cdots ,I\text{,} \end{array}$$

where *x*_*ni*_^*A*^ is the modified input variable and *x*_*ni*_ is the observed input variable, $\left[\max\;\left(f\left(z_{i};{\overset{⌢}{\beta }}^{n}\right)\right)-f\left(z_{i};{\overset{⌢}{\beta }}^{n}\right)\right]$ indicates modification to external environmental variables, and $\left[\max\left({\hat{v}}_{ni}\right)-{\hat{v}}_{ni}\right]$ represents the adjustment of statistical noise.

#### 3.1.3. The Third Stage: The Adjusted Slacks-Based Measure (SBM) Considering Undesirable Output

By replacing the observed input variable *x*_*ni*_ in the first stage with the modified input variables *x*_*ni*_^*A*^ calculated by formula (3), the recalculated efficiency can more properly represent the efficiency of the logistics sector.

When measuring the efficiency of the logistics industry in the 12 provinces of the new western land-sea corridor, the advantages of the three-stage SBM model are as follows: First, by reducing the effects of external environmental variables and random errors and taking into account undesirable output, the third-stage results can more precisely reflect the actual efficiency of DMUs. Second, it is an empirical study on the impact of external environmental variables on efficiency, which can quantify the degree and mechanism of environmental variables.

### 3.2. Malmquist–Luenberger Productivity Index

By replacing the distance function in the Malmquist productivity index with the directional distance function, Chung et al. [25] introduced a Malmquist–Luenberger productivity index that relies on the directional distance function to calculate the total factor productivity of undesirable output, including carbon dioxide emissions.

(4) $$\begin{array}{c} ML_{t}^{t+1}={\left[\frac{\left(1+{\overset{⟶}{D}}_{0}^{t}\left(x^{t},y^{t},b^{t},-b^{t}\right)\right)}{\left(1+{\overset{⟶}{D}}_{0}^{t}\left(x^{t+1},y^{t+1},b^{t+1};y^{t+1},-b^{t+1}\right)\right)}\times \frac{\left(1+{\overset{⟶}{D}}_{0}^{t+1}\left(x^{t},y^{t},b^{t};y^{t},-b^{t}\right)\right)}{\left(1+{\overset{⟶}{D}}_{0}^{t+1}\left(x^{t+1},y^{t+1},b^{t+1};y^{t+1},-b^{t+1}\right)\right)}\right]}^{1/2}, \end{array}$$

where the *ML* productivity index represents the change in DMU's total factor productivity between period *t* and period *t*+1. If *ML* > 1, the total factor productivity rises, if *ML* < 1, the total factor productivity falls, and if *ML*=1, the total factor productivity remains unchanged.

The *ML* productivity index can also be separated into efficiency change index MLEC and technology change index MLTC between period *t* and period *t*+1.

(5) $$\begin{array}{c} ML_{t}^{t+1}=MLEC_{t}^{t+1}\times MLTC_{t}^{t+1}\text{,}\\ MLEC_{t}^{t+1}=\frac{1+{\overset{⟶}{D}}_{0}^{t}\left(x^{t},y^{t},b^{t},-b^{t}\right)}{1+{\overset{⟶}{D}}_{0}^{t+1}\left(x^{t+1},y^{t+1},b^{t+1};y^{t+1},-b^{t+1}\right)}\text{,}\\ MLTC_{t}^{t+1}={\left[\frac{\left\{\left(1\right.+{\overset{⟶}{D}}_{0}^{t+1}\left(x^{t},y^{t},b^{t},-b^{t}\right)\right\}}{\left\{\left(1\right.+{\overset{⟶}{D}}_{0}^{t}\left(x^{t},y^{t},b^{t},-b^{t}\right)\right\}}\times \frac{\left\{1+{\overset{⟶}{D}}_{0}^{t+1}\left(x^{t+1},y^{t+1},b^{t+1};y^{t+1},-b^{t+1}\right)\right\}}{\left\{\left(1\right.+{\overset{⟶}{D}}_{0}^{t}\left(x^{t+1},y^{t+1},b^{t+1};y^{t+1},-b^{t+1}\right)\right\}}\right]}^{1/2}\text{,} \end{array}$$

where MLEC represents efficiency change between period *t* and period *t*+1, MLEC > 1 represents an increase in technical efficiency, MLEC=1 indicates the unchanged technical efficiency, and MLEC < 1 signifies a decline in technological efficiency. MLTC denotes technology transfer between period *t* and period *t*+1, MLTC > 1 represents technical progress, MLTC=1 denotes no technical progress, and MLTC < 1 indicates technical regression.

The efficiency change index MLEC may also be subdivided into two components: the pure technological efficiency change index MLPTEC and the scale efficiency change index MLSEC.

(6) $$\begin{array}{c} ML_{t}^{t+1}=MLEC_{t}^{t+1}\times MLTC_{t}^{t+1}=MLPTEC_{t}^{t+1}\times MLSEC_{t}^{t+1}\times MLTC_{t}^{t+1}\text{.} \end{array}$$

The Malmquist–Luenberger productivity index is actually a modified Malmquist index. The traditional Malmquist index is based on the output distance function, but the Malmquist–Luenberger index is based on the directional distance function, which can improve the good output while reducing the bad output, and the output distance function cannot be realized.

## 4. Indicators and Data

The 2006 China Third Industrial Statistics Yearbook shows that the value added of transport, storage, and postal services account for more than 80 percent of the logistics sector's value added. Therefore, the existing research essentially uses the indicators related to transportation, warehousing, and postal services to represent the logistics industry, and this method has also been adopted in this paper. The input indicators are defined to include capital, labor, and energy consumption, while the output indicators include industry value added and carbon dioxide emissions. Indicators and data processing are described below.

### 4.1. Input Indicators

The fixed asset investment of the whole society in the logistics industry is chosen as the capital indicator, and the capital stock of the logistics industry is calculated by a perpetual inventory system. The formula for calculation is as follows:

(7) $$\begin{array}{c} K_{it}=K_{it-1}\times \left(1-\delta \right)+\frac{I_{it}}{P_{it}}, \end{array}$$

where *K*_it_ and *K*_it−1_ are, respectively, the logistics sector's capital stock in region *i* between *t* and *t* − 1 periods, *K*_*i*0_ is the logistics sector's capital stock in region *i* during the base period, calculated by dividing the amount of fixed assets investment in 2010 by 10% (at 2010 constant price), *δ* is the depreciation rate of capital at 9.6 percent [26], and *I*_it_ and *P*_it_ denote fixed assets investment and fixed assets investment price index in region *i* in period *t*, respectively.

The total number of the logistics sector's urban employees, as well as urban private firms and individuals, is used to calculate the labor force input indicator.

Using the logistics sector's energy consumption as the energy input indicator, converting the various kinds of logistics energy consumption in different provinces into standard coal, and measuring total energy consumption, the following is the formula for processing converted standard coal:

(8) $$\begin{array}{c} E=\overset{11}{\underset{i=1}{\sum }}\left(M_{i}\times P_{i}\right)\text{,} \end{array}$$

where *E* means the total quantity of energy consumption after conversion of all forms of energy consumption to standard coal, *M*_*i*_ represents the various types of energy consumed by the logistics sector, and *P*_*i*_ represents the conversion factor for energy *i* into standard coal.

### 4.2. Output Indicators

The GDP deflator is used to reduce the impact of price variations using the logistics industry's value added as a measure of desirable output indicators, using the base period of 2010. Choosing carbon dioxide emissions of the logistics industry as a measure of undesirable output indicator, carbon dioxide emissions are calculated as the sum of the products of the energy consumption in the logistics industry each year, using the emission factors proposed in 2006 by the United Nations Intergovernmental Panel on Climate Change (IPCC).

### 4.3. External Environmental Variables

External environmental variables primarily comprise aspects that have a considerable influence on the efficiency of the logistics sector but are beyond the control of the logistics industry itself. In this paper, the elements of the external environment are selected from four categories: economic condition, informatization development, industrial market scale, and import and export.

First, the provincial GDP is selected as a measure of economic condition and processed through the GDP deflator. The improvement of provincial economic conditions has a favorable influence on the development of the logistics sector as well as the efficiency of the logistics industry. Second, the number of mobile phone users at year-end in each province has been chosen as an essential indicator to assess the level of development of information technology. The popularity of smartphones makes information more accessible, and the terminal development of logistics information systems shifts to mobile, driving the growth of the logistics sector and influencing logistics sector efficiency. Third, the industry market scale, the continuous optimization of the industrial market size has led to the fast expansion of the logistics sector, which has had a positive influence on the efficiency of the logistics industry, and the total number of registered legal entities in the logistics business in each province is a key measure for assessing the industry's growth. Fourth, the total import and export in each province is chosen as the import and export measurement, which assists its logistics industry in opening up international markets and promoting the integration of domestic and foreign commodities' markets.

### 4.4. Data Sources

This paper examines the logistics sector in 12 provinces along the new western land-sea corridor between 2010 and 2019, covering inner Mongolia, Guangxi, Hainan, Chongqing, Sichuan, Guizhou, Yunnan, Shaanxi, Gansu, Qinghai, Ningxia, and Xinjiang (Tibet is not included due to missing data on energy consumption). Data from transportation, storage, and postal services are used to replace the statistics of the logistics industry. The collected data is from the websites of the China National Bureau of Statistics, the China Energy Statistics Yearbook, and the China Statistics Yearbook.  Table 1 displays the descriptive data for critical factors.

In order to make the measurement result more reasonable, the Pearson's correlation test of input-output indicators is carried out by using Stata 16. The correlation coefficient of input and output indicators is high, all of which passed the 1% significance test and satisfied isotropy requirements; Table 2 displays the results.

## 5. Empirical Results

### 5.1. Three-Stage SBM with Undesirable Output

#### 5.1.1. The First Stage

The initial input and output data from the logistics business from 2010 to 2019 were substituted into the input-oriented SBM model utilizing 12 provinces as DMUs, and technical efficiency, pure technical efficiency, and scale efficiency in the logistics sector were derived using the MaxDEA Pro8 software, with the results shown in Tables 3–5.

Overall, the average technical efficiency of the logistics sector increased from 0.657 in 2010 to 0.695 in 2019, while the average pure technical efficiency climbed from 0.785 in 2010 to 0.823 in 2019, and the average scale efficiency increased from 0.834 in 2010 to 0.866 in 2019 across 12 provinces, which has not yet reached the production frontier. It is suggested that although the technical efficiency of the logistics sector has improved in the provinces along the new western land-sea corridor, it is still usually low and its growth is slow. By area, the logistics sector's average technical efficiency is higher in the northern area than in the southern area of the corridor, with the northern area decreasing from 0.792 in 2010 to 0.76 in 2019 and the southern area increasing from 0.522 in 2010 to 0.629 in 2019. By province, the logistics sector efficiency varies substantially among provinces, and the unbalanced growth of the logistics industry is quite prominent. While insisting on the expansion of the logistics sector, some provinces place a premium on environmental preservation and are able to approach the production frontier in terms of technical efficiency, while others have more opportunity for efficiency improvement in general. Ningxia, Inner Mongolia, and Shaanxi are the top three provinces in terms of average technical efficiency, all around 0.9, implying that these provinces are close to the production frontier. Sichuan, Qinghai, and Hainan have the lowest technical efficiency in logistics industry, of which Sichuan is 0.532. The technical efficiency of the logistics sector in Sichuan increased from 0.386 in 2010 to 0.726 in 2017 and decreased to 0.554 in 2019. From 2014 to 2019, pure technical efficiency was at the forefront of production, but scale efficiency continued to decline, leading to a decrease in technical efficiency. The logistics industry's technical efficiency in Qinghai has been on a slow downward trend except for a slight increase in 2015. Although the pure technical efficiency was at the production frontier, scale efficiency fluctuated around 0.5 percent, which led to a decline of technical efficiency. In the Hainan's logistics business, the trend of technical efficiency was more consistent with pure technical efficiency, and the increase of scale efficiency results in the fluctuation of technical efficiency. The logistics sector in Guangxi, Chongqing, Guizhou, Yunnan, Gansu, and Xinjiang was less technologically efficient overall, but the scale efficiency was high and the pure technical efficiency was low, which led to low technical efficiency.

#### 5.1.2. The Second Stage

In the Stochastic frontier analysis (SFA), explanatory variables are the input slack variables obtained in the first phase, economic development, informatization development, industry market scale, and import and export are the independent variables, while the frontier 4.1 software can be used to study the impact of external environmental factors on the input slack variables, as detailed in Table 6.

Table 6 demonstrates that the one-sided likelihood ratio tests are 34.03, 31.77, and 57.28, respectively, all of which are significantly tested at a level of 1%. It suggests that external environmental variables should be excluded when studying the technical efficiency of the logistics sector along the new western land-sea corridor, and the estimation result of the SFA model is acceptable. All three gamma values passed the significance test of 1%, which shows that the selected external environmental variables are more plausible. When the external environmental variables are positively correlated with the input slack variables, it means that increasing the external environmental variables will increase input redundancy and decrease technical efficiency. When the external environmental variables are negatively correlated with the input slack variables, reducing the external environmental variables helps to minimize input redundancy and increase the logistics sector's technical efficiency. With the provincial gross domestic product (GDP), the number of mobile phone users at year-end, the number of registered legal entities in the logistics business, and the provincial total imports and exports employed as explanatory variables, most of the variables passed the 1% level significance test.

*(1) Economic Condition*. The provincial gross domestic product (GDP) is a measure of economic growth, which is negatively related to three slack elements. It implies that the improvement of economic conditions can reduce the input redundancy of capital stock and employees' energy consumption, reasonably allocate the resources of the logistics industry, and improve technical efficiency in the logistics industry.

*(2) Informatization Development*. The informatization level represented by the number of mobile phone users at year-end shows a substantial positive connection with the slack variables of capital stock and energy consumption and a significant negative correlation with the slack variables of employees, all of which pass the 1 percentage point significance test. This suggests that the increase in mobile phone users at year-end will boost the redundancy of capital stock and energy consumption inputs, which will lead to inefficiencies in capital inputs and energy consumption, while reducing the redundancy of employee inputs to make them more rational.

*(3) Industry Market Scale*. The industry market scale represented by the number of registered legal entities throughout the logistics business has a high positive association with energy consumption slack variables, a negative correlation with capital slack variables, and no significant relationship with employee slack variables. This shows that as the number of registered legal persons increases, so will the number of firms, resulting in lower energy efficiency and more rational capital allocation.

*(4) Import and Export*. The provincial total imports and exports are significantly positively correlated with slack variables of employee and energy consumption, but negligible with capital stock. It implies that an increase in import and export will generate redundancy in the number of employees and energy consumption, causing irrational input of employees and inefficient use of energy in the logistics industry.

#### 5.1.3. The Third Stage

The SBM model was applied to calculate the adjusted input variables instead of observed input variables to obtain accurate technical efficiency, pure technical efficiency, and scale efficiency in the logistics industry, removing the impacts of environmental factors and statistical noise, as illustrated in Tables 7–9.

Overall, the average technical efficiency in the logistics sector increased from 0.710 in the first phase to 0.734 in the third phase in 12 provinces along the new western land-sea corridor, indicating that, despite a lower average technical efficiency, uncertainties such as external environment variables continue to underestimate the logistics industry's technical efficiency. The average technical efficiency of the logistics sector in the southern area increased from 0.635 in the first phase to 0.783 in the third phase, and the logistics sector's average technical efficiency in the northern area decreased from 0.786 in the first phase to 0.715 in the third phase, indicating the adjusted average technical efficiency in the southern area is higher.

Technical efficiency in the logistics sector varies widely among provinces, both before and after adjustments. The average technical efficiency of Guangxi's logistics industry rose from 0.656 in the first step to 0.904 in the third step, and that of Chongqing's logistics industry rose from 0.685 in the first step to 0.917 in the third step, both of which showed that external environment variables had a great influence. Among them, improving the pure technical efficiency seems to be the key factor for improving the logistics sector's technical efficiency in Guangxi and Chongqing, and increasing the logistics sector's scale efficiency can only affect the technical efficiency in Chongqing. Inner Mongolia and Shaanxi have much higher efficiency levels in the logistics industry than other provinces. Inner Mongolia's adjusted technical efficiency reached the production frontier, and Shaanxi's adjusted technical efficiency was 0.969, mainly because Inner Mongolia and Shaanxi are close to central China, with relatively good transportation infrastructure conditions, relatively large labor and capital investment. The logistic industry's technical efficiency in Qinghai and Ningxia declined from 0.544 to 0.961 in the first step to 0.259 and 0.697 in the third step, respectively. The two provinces' pure technical efficiency is at the production frontier. The decline in technical efficiency is mainly due to a fall in scale efficiency, demonstrating that the high efficiency of the first step is influenced by changes in the external environment. Although pure technical efficiency has improved in Hainan, Guizhou, Gansu, and Xinjiang, scale efficiency has decreased, resulting in a slight decrease in the logistics industry's technical efficiency, indicating that external environmental variables have not significantly driven the logistics industry's development.

#### 5.1.4. Malmquist–Luenberger Productivity Index

This paper uses MaxDEA Pro8 to substitute the adjusted input and initial output variables into the Malmquist–Luenberger productivity index to calculate the changes of total factor productivity in 12 provinces along the new western land-sea corridor from 2010 to 2019, and the calculation results are shown in Tables 10 and 11.

The Malmquist–Luenberger productivity index remained higher than 1 except in 2015–2016, 2016–2017, and 2018–2019. Over the last decade, the Malmquist–Luenberger productivity index for logistics businesses along the new western land-sea corridor has averaged 1.048, which indicates that the total factor productivity is increasing and that the logistics industry is developing quicker. On average, the technical change index increased by 6.6 percent, but the efficiency change index decreased by 1.5 percent. Because the efficiency change index has declined at a slower rate than the technical change index, the average annual growth of TFP has remained at 4.8 percent over the past decade, suggesting that technological progress is a key factor in increasing TFP. The scale efficiency change contributed −1.6 percent to total factor productivity index change, indicating that change in the scale efficiency has a detrimental impact on total factor productivity improvement. The efficiency change index was less than 1 in 7 out of 10 years, and the lowest being 0.937 in 2018–2019, indicating a downward trend. However, the technical change index was greater than 1 in 7 out of 10 years, and the highest value was 1.199 in 2014–2015, indicating an upward trend. Furthermore, the Malmquist–Luenberger index and the technical change index kept the same overall trends, with an apparent upward trend only in 2014–2015.

Only Qinghai had a Malmquist–Luenberger productivity index less than 1 among the 12 provinces, while the rest provinces had a Malmquist–Luenberger productivity index more than 1. The average Malmquist–Luenberger productivity index was 1.049, indicating an overall increase in the total factor productivity, with 92 percent of provinces contributing to an increase in the logistics industry's total factor productivity. Technical change indexes of all provinces were greater than 1, with an average of 1.070, indicating an overall upward trend in the total factor productivity in the logistics sector. The pure technical efficiency change index was less than 1 in 5 provinces and greater than 1 in 7 provinces. The overall mean of the pure technical efficiency change index was 1.003, indicating an upward trend in 58.3 percent of the provinces in the logistics sector. The average Malmquist–Luenberger index, as well as the average index of technical change in the southern and northern areas, were both more than 1, whereas the average index of scale efficiency change was less than 1. The acceleration of technological advancement is the reason for the growth of total factor productivity in the logistics sector in the 12 provinces of the new western land-sea corridor, and the primary decrease is the fall in scale efficiency.

## 6. Conclusions and Policy Proposals

This article considers the relationship between logistics sector expansion and environmental protection in a systematic manner, using panel data from the logistics industry along China's new western land-sea corridor between 2010 and 2019, and measures actual logistics industry efficiency after excluding the impact of external environmental variables as well as statistical noise by employing nonradial, nonoriented three-stage SBM with undesirable output. Finally, the Malmquist–Luenberger productivity index is used to study the dynamic evolution of logistics business efficiency, and the following conclusions are drawn:

1. External environmental variables have a great influence on the efficiency of the logistics sector. Economic conditions, informatization development, industrial market scale, and import and export all have an influence on the logistics sector's efficiency. The efficiency of the logistics business varies between the first and third phases, and the effect of each external environment variable on the logistics sector efficiency is different.
2. In general, the overall logistics sector efficiency in the new western land-sea corridor remains low, despite ongoing improvement. The logistics industry's resource allocation is insufficiently optimized, and the development rate is rather modest. The pure technical efficiency is relatively high, and it is the key factor influencing the expansion of the technical efficiency, while the scale of the logistics sector does not correspond to the current level of industrial development.
3. The technical efficiency in the logistics sector in the southern and northern areas of the new western land-sea corridor both have development potential. On average, the logistics industry's technical efficiency in the southern area is greater than that in the northern area, while it is substantially higher in the provinces near central China than in the remote hinterland areas.
4. The efficiency of the logistics business varies greatly by province. Except for Inner Mongolia, where the adjusted efficiency of the logistics sector is on the production frontier, the technical efficiency of other provinces has changed significantly in the past 10 years. Shaanxi and Chongqing continue to have the highest adjusted technical efficiency, while Qinghai, Xinjiang, and Hainan have the lowest.
5. Over the 10 year period, the total factor productivity of the logistics industry along the new western land-sea corridor has improved by approximately 4.8 percent each year, while the technological change index increased by an average of 6.6 percent every year, indicating an overall improvement. The primary cause of the improvement is technical development, whereas the primary cause of the drop is the decrease in scale efficiency. The total factor productivity of the logistics industry in 92% of the provinces in the new western land-sea corridor has improved.

This research makes the following recommendations relying on the measurement results:

Firstly, it is essential to continually improve the external environment in order to help the expansion of the logistics firms. Given the variety of external environmental variables in each province along the new western land-sea corridor, environmental adjustments have resulted in significant variances in logistics sector efficiency in various provinces. Each province should pool its resources and develop regulations to increase logistics business efficiency, as well as encourage logistics enterprises to grow larger and stronger through government investment, form a market operation mode guided by the government but dominated by enterprises, and accelerate resource gathering.

Secondly, it is necessary to enhance both pure technical efficiency and scale efficiency. The technical efficiency is mostly governed by the pure technical efficiency of the logistics sector in each province, and the average scale efficiency of most provinces is declining. Each province should take full advantage of the opportunity of “new infrastructure” construction, upgrade and promote logistics information technology and the connection between railway freight transport and port hubs, promote the construction of a perfect multimodal transport system and enhance air-rail and other modes of transportation, integrate cargo capacity with Internet platforms, and promote cross-regional cooperation in the logistics industry.

Thirdly, it is crucial to enhance the current operating efficiency of the new western land-sea corridor to launch the new western land-sea corridor's close connection with the Yangtze River Economic Belt, ensure smooth southbound rail-sea and international railway intermodal transport, strengthen synergistic and joint development inside and outside the corridor, and encourage low costs and service enhancement in the logistics sector.

## Figures and Tables

**Figure 1:** The research frameworks.

**Table 1:** Descriptive statistics.

Indicator type	Indicator name	Sample	Average	Standard deviation	Minimum	Maximum
Input	Logistics industry total social fixed asset investment (100 million yuan)	120	7893.046	5676.191	1188.355	29314.7
	Logistics industry urban employment (10,000 people)	120	342.8625	259.7919	46.5	1175.5
	Logistics industry energy consumption (10,000 tons of standard coal)	120	728.7934	391.618	110.7651	1715.842

Desirable output	Logistics industry value added (100 million yuan)	120	533.1633	330.8203	70.7	1473.1

Undesirable output	Carbon dioxide emissions from logistics industry (10,000 tons)	120	1793.214	958.1894	285.3466	4083.725

External environmental variables	Economic condition (100 million yuan)	120	10829.42	8099.973	1144.2	43169.27
	Informatization development (10,000 households)	120	2670.013	1800.94	290.3	9443.5
	Industrial market scale (units)	120	5623.533	4161.654	471	19283
	Import and export (US $100 million)	120	241.013	235.7846	5.44815	984.0066

**Table 2:** Pearson's correlation coefficient of logistics industry input-output indicators.

Input-output indicators	Total social fixed asset investment	Urban employment	Energy consumption
Value added	0.8728^*∗∗∗*^	0.8149^*∗∗∗*^	0.8738^*∗∗∗*^
Carbon dioxide emissions	0.8701^*∗∗∗*^	0.7124^*∗∗∗*^	0.9983^*∗∗∗*^

*Note.* ^*∗∗∗*^indicates significance at 1% level.

**Table 3:** Logistics industry's technical efficiency in the first stage of the new western land-sea corridor.

Province	2010	2011	2012	2013	2014	2015	2016	2017	2018	2019	Average
Inner Mongolia	0.744	1.000	1.000	0.681	0.747	0.959	1.000	1.000	1.000	1.000	0.913
Guangxi	0.571	0.627	0.586	0.630	0.660	0.772	0.733	0.725	0.653	0.602	0.656
Hainan	0.443	0.458	0.456	0.450	0.532	0.652	0.717	0.716	0.662	0.722	0.581
Chongqing	0.766	0.769	0.629	0.601	0.677	0.698	0.728	0.680	0.665	0.635	0.685
Sichuan	0.386	0.411	0.378	0.472	0.554	0.573	0.574	0.726	0.690	0.554	0.532
Guizhou	0.606	0.736	0.607	0.578	0.677	0.829	1.000	1.000	0.728	0.640	0.740
Yunnan	0.356	0.380	0.409	0.449	0.518	1.000	0.868	0.829	0.721	0.621	0.615
Shaanxi	1.000	0.757	0.732	0.706	0.821	1.000	1.000	0.984	0.813	0.741	0.855
Gansu	1.000	1.000	0.878	0.750	0.734	0.765	0.742	0.732	0.701	0.661	0.796
Qinghai	0.569	0.599	0.563	0.528	0.599	0.643	0.576	0.528	0.437	0.394	0.544
Ningxia	1.000	1.000	1.000	1.000	1.000	1.000	1.000	1.000	0.845	0.766	0.961
Xinjiang	0.439	0.453	0.504	0.484	0.618	0.668	0.695	0.589	1.000	1.000	0.645
Average	0.657	0.682	0.645	0.611	0.678	0.797	0.803	0.793	0.743	0.695	0.710
Southern area average	0.522	0.563	0.511	0.530	0.603	0.754	0.770	0.779	0.687	0.629	0.635
Northern area average	0.792	0.801	0.780	0.691	0.753	0.839	0.835	0.806	0.799	0.760	0.786

**Table 4:** Logistics industry's pure technical efficiency in the first stage of the new western land-sea corridor.

Province	2010	2011	2012	2013	2014	2015	2016	2017	2018	2019	Average
Inner Mongolia	1.000	1.000	1.000	1.000	1.000	1.000	1.000	1.000	1.000	1.000	1.000
Guangxi	0.717	0.811	0.773	0.863	0.789	0.824	0.737	0.736	0.660	0.613	0.752
Hainan	0.619	0.631	0.639	0.609	0.651	0.673	0.740	0.826	0.744	0.857	0.699
Chongqing	1.000	1.000	1.000	1.000	0.821	0.764	0.729	0.687	0.670	0.642	0.831
Sichuan	0.500	0.530	0.507	0.629	1.000	1.000	1.000	1.000	1.000	1.000	0.817
Guizhou	0.674	0.774	0.706	0.754	1.000	0.845	1.000	1.000	0.746	0.668	0.817
Yunnan	0.432	0.447	0.524	0.613	0.620	1.000	0.869	0.835	0.723	0.624	0.669
Shaanxi	1.000	1.000	1.000	1.000	1.000	1.000	1.000	1.000	0.815	0.744	0.956
Gansu	1.000	1.000	1.000	1.000	1.000	0.814	0.754	0.785	0.740	0.723	0.882
Qinghai	1.000	1.000	1.000	1.000	1.000	1.000	1.000	1.000	0.721	1.000	0.972
Ningxia	1.000	1.000	1.000	1.000	1.000	1.000	1.000	1.000	1.000	1.000	1.000
Xinjiang	0.479	0.468	0.566	0.614	0.725	0.722	0.699	0.606	1.000	1.000	0.688
Average	0.785	0.805	0.810	0.840	0.884	0.887	0.877	0.873	0.818	0.823	0.840
Southern area average	0.657	0.699	0.691	0.745	0.813	0.851	0.846	0.847	0.757	0.734	0.764
Northern area average	0.913	0.911	0.928	0.936	0.954	0.923	0.909	0.899	0.879	0.911	0.916

**Table 5:** Logistics industry's scale efficiency in the first stage of the new western land-sea corridor.

Province	2010	2011	2012	2013	2014	2015	2016	2017	2018	2019	Average
Inner Mongolia	0.744	1.000	1.000	0.681	0.747	0.959	1.000	1.000	1.000	1.000	0.913
	Drs	—	—	Drs	Drs	Drs	—	—	—	—	

Guangxi	0.797	0.773	0.759	0.731	0.837	0.937	0.995	0.985	0.990	0.982	0.879
	Drs	Drs	Drs	Drs	Drs	Drs	Irs	Irs	Irs	Irs	

Hainan	0.716	0.726	0.714	0.739	0.817	0.968	0.969	0.867	0.890	0.842	0.825
	Irs	Irs	Irs	Irs	Irs	Irs	Irs	Irs	Irs	Irs	

Chongqing	0.766	0.769	0.629	0.601	0.825	0.914	0.999	0.989	0.992	0.990	0.847
	Drs	Drs	Drs	Drs	Drs	Drs	Irs	Irs	Irs	Irs	

Sichuan	0.773	0.775	0.745	0.750	0.554	0.573	0.574	0.726	0.690	0.554	0.671
	Drs	Drs	Drs	Drs	Drs	Drs	Drs	Drs	Drs	Drs	

Guizhou	0.899	0.951	0.859	0.768	0.677	0.981	1.000	1.000	0.975	0.958	0.907
	Drs	Drs	Drs	Drs	Drs	Drs	—	—	Irs	Irs	

Yunnan	0.824	0.851	0.781	0.732	0.836	1.000	0.999	0.993	0.997	0.994	0.901
	Drs	Drs	Drs	Drs	Drs	—	Irs	Irs	Irs	Irs	

Shaanxi	1.000	0.757	0.732	0.706	0.821	1.000	1.000	0.984	0.997	0.996	0.899
	—	Drs	Drs	Drs	Drs	—	—	Drs	Irs	Irs	

Gansu	1.000	1.000	0.878	0.750	0.734	0.941	0.983	0.932	0.947	0.914	0.908
	—	—	Drs	Drs	Drs	Drs	Irs	Irs	Irs	Irs	

Qinghai	0.569	0.599	0.563	0.528	0.599	0.643	0.576	0.528	0.606	0.394	0.560
	Irs	Irs	Irs	Irs	Irs	Irs	Irs	Irs	Irs	Irs	

Ningxia	1.000	1.000	1.000	1.000	1.000	1.000	1.000	1.000	0.845	0.766	0.961
	—	—	—	—	—	—	—	—	Irs	Irs	

Xinjiang	0.916	0.968	0.890	0.788	0.852	0.926	0.995	0.972	1.000	1.000	0.931
	Drs	Drs	Drs	Drs	Drs	Drs	Irs	Irs	—	—	

Average	0.834	0.847	0.796	0.731	0.775	0.903	0.924	0.915	0.911	0.866	0.850

Southern area average	0.796	0.808	0.748	0.720	0.758	0.895	0.923	0.927	0.922	0.887	0.838

Northern area average	0.871	0.887	0.844	0.742	0.792	0.911	0.926	0.903	0.899	0.845	0.862

*Note.* irs, drs, and “—” represent increasing, decreasing, and constant returns to scale, respectively.

**Table 6:** Second stage for SFA regression results.

Variable	Capital stock slack variable		Employee slack variable		Energy consumption slack variable	
	Coefficient	*t* value	Coefficient	*t* value	Coefficient	*t* value
Constant term	−550.08	−1.58	12.75	0.90	8.63	0.50
Economic condition	−12170.524^*∗∗∗*^	−15.18	−421.26^*∗*^	−1.74	−2824.50^*∗∗∗*^	−6.70
Informatization development	78220.576^*∗∗∗*^	177.01	−599.99^*∗∗∗*^	−2.74	2161.98^*∗∗∗*^	5.13
Industry market scale	−1778.34^*∗∗∗*^	−4.29	−415.43	−0.71	3468.94^*∗∗∗*^	4.95
Import and export	296.32	0.34	415.7825^*∗∗∗*^	6.41	231.79^*∗∗∗*^	3.01
Sigma-squared	6601762.70^*∗∗∗*^	2627652.00	13050.99^*∗∗∗*^	66.78	36212.30^*∗∗∗*^	6556.07
Gamma	0.53^*∗∗∗*^	7.65	0.58^*∗∗∗*^	10.71	0.73^*∗∗∗*^	20.83

Log likelihood function	−1076.76		−717.98		−740.05	
One-sided likelihood ratio test	34.03^*∗∗∗*^		31.77^*∗∗∗*^		57.28^*∗∗∗*^	

*Note.* ^*∗*^, ^*∗∗*^, and ^*∗∗∗*^ are significant at 10%, 5%, and 1%, respectively.

**Table 7:** Logistics industry's technical efficiency in the third stage of the new western land-sea corridor.

Province	2010	2011	2012	2013	2014	2015	2016	2017	2018	2019	Average
Inner Mongolia	1.000	1.000	1.000	1.000	1.000	1.000	1.000	1.000	1.000	1.000	1.000
Guangxi	0.906	0.920	0.920	1.000	0.915	0.940	0.885	0.875	0.855	0.823	0.904
Hainan	0.367	0.361	0.378	0.377	0.400	0.480	0.453	0.412	0.391	0.386	0.401
Chongqing	1.000	1.000	1.000	0.901	1.000	0.942	0.862	0.828	0.827	0.812	0.917
Sichuan	0.789	0.783	0.795	0.863	0.783	0.698	0.672	1.000	0.823	0.716	0.792
Guizhou	0.700	0.720	0.742	0.724	0.675	0.741	0.649	0.672	0.724	0.692	0.704
Yunnan	0.679	0.694	0.757	0.778	0.814	0.835	0.818	0.864	0.879	0.831	0.795
Shaanxi	1.000	0.964	1.000	1.000	1.000	1.000	1.000	0.914	0.934	0.883	0.969
Gansu	0.788	0.798	1.000	0.701	0.666	0.700	0.630	0.599	0.579	0.550	0.701
Qinghai	0.293	0.279	0.282	0.276	0.270	0.281	0.256	0.237	0.227	0.184	0.259
Ningxia	1.000	1.000	1.000	1.000	1.000	0.513	0.463	0.373	0.325	0.293	0.697
Xinjiang	0.584	0.581	0.679	0.631	0.725	0.729	0.680	0.639	0.728	0.677	0.665
Average	0.759	0.758	0.796	0.771	0.771	0.738	0.697	0.701	0.691	0.654	0.734
Southern area average	0.777	0.777	0.799	0.806	0.798	0.805	0.763	0.795	0.776	0.735	0.783
Northern area average	0.778	0.770	0.827	0.768	0.777	0.704	0.672	0.627	0.632	0.598	0.715

**Table 8:** Logistics industry's pure technical efficiency in the third stage of the new western land-sea corridor.

Province	2010	2011	2012	2013	2014	2015	2016	2017	2018	2019	Average
Inner Mongolia	1.000	1.000	1.000	1.000	1.000	1.000	1.000	1.000	1.000	1.000	1.000
Guangxi	0.956	0.960	1.000	1.000	1.000	1.000	0.971	0.978	0.953	0.940	0.976
Hainan	0.946	1.000	1.000	0.965	0.975	0.970	0.974	0.985	0.976	1.000	0.979
Chongqing	1.000	1.000	1.000	1.000	1.000	0.971	0.926	0.913	0.906	0.891	0.961
Sichuan	0.791	0.799	0.826	0.894	1.000	1.000	1.000	1.000	1.000	1.000	0.931
Guizhou	0.939	0.948	0.936	0.948	1.000	0.960	1.000	1.000	0.924	0.900	0.955
Yunnan	0.788	0.794	0.856	0.896	0.881	1.000	1.000	1.000	0.908	0.864	0.899
Shaanxi	1.000	1.000	1.000	1.000	1.000	1.000	1.000	0.952	0.969	0.916	0.984
Gansu	1.000	1.000	1.000	1.000	1.000	1.000	0.959	1.000	0.970	0.956	0.989
Qinghai	1.000	1.000	1.000	1.000	1.000	1.000	1.000	1.000	0.968	1.000	0.997
Ningxia	1.000	1.000	1.000	1.000	1.000	1.000	1.000	1.000	1.000	1.000	1.000
Xinjiang	0.889	0.898	0.922	0.913	0.935	0.907	0.899	0.846	1.000	1.000	0.921
Average	0.942	0.950	0.962	0.968	0.983	0.984	0.977	0.973	0.965	0.956	0.966
Southern area average	0.903	0.917	0.936	0.950	0.976	0.984	0.979	0.979	0.945	0.933	0.950
Northern area average	0.981	0.983	0.987	0.985	0.989	0.985	0.976	0.966	0.985	0.979	0.982

**Table 9:** Logistics industry's scale efficiency in the third stage of the new western land-sea corridor.

Province	2010	2011	2012	2013	2014	2015	2016	2017	2018	2019	Average
Inner Mongolia	1.000	1.000	1.000	1.000	1.000	1.000	1.000	1.000	1.000	1.000	1.000
	—	—	—	—	—	—	—	—	—	—	

Guangxi	0.948	0.959	0.920	1.000	0.915	0.940	0.911	0.894	0.897	0.875	0.926
	Irs	Irs	Irs	—	Irs	Irs	Irs	Irs	Irs	Irs	

Hainan	0.388	0.361	0.378	0.391	0.410	0.495	0.465	0.419	0.401	0.386	0.409
	Irs	Irs	Irs	Irs	Irs	Irs	Irs	Irs	Irs	Irs	

Chongqing	1.000	1.000	1.000	0.901	1.000	0.970	0.930	0.907	0.913	0.912	0.953
	—	—	—	Irs	—	Irs	Irs	Irs	Irs	Irs	

Sichuan	0.996	0.980	0.962	0.966	0.783	0.698	0.672	1.000	0.823	0.716	0.860
	Irs	Irs	Irs	Irs	Drs	Drs	Drs	—	Drs	Drs	

Guizhou	0.746	0.759	0.793	0.764	0.675	0.772	0.649	0.672	0.784	0.769	0.738
	Irs	Irs	Irs	Irs	Irs	Irs	Irs	Irs	Irs	Irs	

Yunnan	0.862	0.873	0.884	0.869	0.924	0.835	0.818	0.864	0.968	0.961	0.886
	Irs	Irs	Irs	Irs	Irs	Irs	Irs	Irs	Irs	Irs	

Shaanxi	1.000	0.964	1.000	1.000	1.000	1.000	1.000	0.959	0.964	0.964	0.985
	—	Irs	—	—	—	—	—	Irs	Irs	Irs	

Gansu	0.788	0.798	1.000	0.701	0.666	0.700	0.657	0.599	0.597	0.575	0.708
	Irs	Irs	—	Irs	Irs	Irs	Irs	Irs	Irs	Irs	

Qinghai	0.293	0.279	0.282	0.276	0.270	0.281	0.256	0.237	0.235	0.184	0.259
	Irs	Irs	Irs	Irs	Irs	Irs	Irs	Irs	Irs	Irs	

Ningxia	1.000	1.000	1.000	1.000	1.000	0.513	0.463	0.373	0.325	0.293	0.697
	—	—	—	—	—	Irs	Irs	Irs	Irs	Irs	

Xinjiang	0.657	0.646	0.736	0.692	0.776	0.804	0.757	0.755	0.728	0.677	0.723
	Irs	Irs	Irs	Irs	Irs	Irs	Irs	Irs	Irs	Irs	

Average	0.807	0.802	0.830	0.797	0.785	0.751	0.715	0.723	0.720	0.693	0.762

Southern area average	0.823	0.822	0.823	0.815	0.785	0.785	0.741	0.793	0.798	0.770	0.795

Northern area average	0.790	0.781	0.836	0.778	0.785	0.716	0.689	0.654	0.641	0.616	0.729

*Note.* irs, drs, and “—” represent increasing, decreasing and constant returns to scale, respectively.

**Table 10:** Malmquist–Luenberger productivity index of logistics industry in the new western land-sea corridor.

Year	Efficiency change index	Technical change index	Pure technical efficiency change index	Scale efficiency change index	Malmquist–Luenberger productivity index
2010-2011	0.997	1.178	1.008	0.989	1.175
2011-2012	1.054	0.958	1.014	1.040	1.007
2012-2013	0.974	1.104	1.008	0.966	1.074
2013-2014	1.004	1.077	1.016	0.990	1.083
2014-2015	0.983	1.199	1.003	0.982	1.157
2015-2016	0.939	1.046	0.993	0.945	0.981
2016-2017	0.998	0.995	0.995	1.003	0.994
2017-2018	0.983	1.040	0.994	0.992	1.022
2018-2019	0.937	0.999	0.990	0.947	0.936
Average	0.985	1.066	1.002	0.984	1.048

**Table 11:** Malmquist–Luenberger productivity index of logistics industry in 12 provinces in the new western land-sea corridor.

Provinces	Efficiency change index	Technical change index	Pure technical efficiency change index	Scale efficiency change index	Malmquist–luenberger productivity index
Inner Mongolia	1.000	1.029	1.000	1.000	1.029
Guangxi	0.991	1.050	0.998	0.992	1.041
Hainan	1.009	1.039	1.006	1.003	1.049
Chongqing	0.979	1.076	0.987	0.991	1.054
Sichuan	1.004	1.063	1.027	0.979	1.065
Guizhou	1.001	1.039	0.996	1.009	1.040
Yunnan	1.023	1.047	1.012	1.014	1.073
Shaanxi	0.987	1.121	0.991	0.996	1.108
Gansu	0.970	1.089	0.995	0.975	1.046
Qinghai	0.952	1.038	1.000	0.952	0.989
Ningxia	0.888	1.149	1.000	0.888	1.001
Xinjiang	1.021	1.055	1.015	1.006	1.079
Average	1.001	1.052	1.005	0.998	1.054
Southern area average	0.970	1.080	1.000	0.970	1.042
Northern area average	0.984	1.070	1.003	0.982	1.049

## Data Availability

The experimental data used to support the findings of this study are available from the corresponding author upon request.
